# Wind Tunnel Analysis of the Aerodynamic Loads on Rolling Stock over Railway Embankments: The Effect of Shelter Windbreaks

**DOI:** 10.1155/2014/421829

**Published:** 2014-11-12

**Authors:** Sergio Avila-Sanchez, Santiago Pindado, Oscar Lopez-Garcia, Angel Sanz-Andres

**Affiliations:** ^1^Instituto Universitario de Microgravedad “Ignacio Da Riva” (IDR/UPM), Universidad Politécnica de Madrid, ETSI Aeronáutica y del Espacio, Plaza del Cardenal Cisneros 3, 28040 Madrid, Spain; ^2^Departamento de Aeronaves y Vehículos Espaciales, Universidad Politécnica de Madrid, ETSI Aeronáutica y del Espacio, Plaza del Cardenal Cisneros 3, 28040 Madrid, Spain

## Abstract

Wind-flow pattern over embankments involves an overexposure of the rolling stock travelling on them to wind loads. Windbreaks are a common solution for changing the flow characteristic in order to decrease unwanted effects induced by the presence of cross-wind. The shelter effectiveness of a set of windbreaks placed over a railway twin-track embankment is experimentally analysed. A set of two-dimensional wind tunnel tests are undertaken and results corresponding to pressure tap measurements over a section of a typical high-speed train are herein presented. The results indicate that even small-height windbreaks provide sheltering effects to the vehicles. Also, eaves located at the windbreak tips seem to improve their sheltering effect.

## 1. Introduction

### 1.1. Effect of Embankments on the Wind-Flow Profile

Although the wind effects on certain human activities such as farming or city planning have been well known throughout history (see, for instance,* De Agri Cultura* by Marcus Porcius Cato—also known as Cato the Elder—, and* De Architectura Libri Decem* by Marcus Vitruvius Pollio [1, 2]), it could be said that the effect of the wind on structures and constructions only started to be rationally studied in the XIX century. There are many works in the literature devoted to analysing the interaction between wind and civil engineering structures [3–5]. The efforts to increase the safety of constructions have resulted in standard codes, which classify the wind effects as a function of the local terrain, establishing the maximum loads on a reduced number of typical building forms [6, 7]. The acceleration of the wind in the surroundings of hills is normally the object of special attention in the aforementioned standard codes, as both the increase of wind speed and the change of its direction can produce high wind loads on elements located there [8–11]. More specifically, the wind-flow pattern on railway embankments represents a good example of this problem, as it could significantly increase the wind loads on rolling stocks and, therefore, the risk of overturning [12–17]. In addition, taking into account the work by Kim et al. [18] it can also be noted that changes on the wind-flow pattern due to artificial structures erected on the terrain of a specific location can produce not only higher wind loads, but also temperature variations that could lead to negative effects on crop yields. Moreover, these authors clearly state that “highway embankments influence the lower currents at the bottom of a slope” and “there have not been sufficient studies carried out on airflow near an artificial structure such as a highway embankment.”

### 1.2. Reduction on Wind Action by Using Shelters/Parapets/Screens

One of the most effective ways to reduce the wind effects is by placing screens or windbreaks, either solid or porous, upstream the elements to be protected. Unfortunately, these specific elements produce new flow patterns due to wake interactions or, more directly, due to changes in the flow velocity distribution that could lead to the introduction of additional wind loads. As an example, the fences formed by trees and bushes have been traditionally used in agriculture to protect crops [19–22], the use of this kind of windbreaks being spread throughout the XX century to other applications such as odour dispersion [23] or noise reduction [24]. After some former studies in this field [25, 26], several research works have been carried out at the IDR/UPM Institute to analyse the effectiveness of parapets in alleviating wind effects on different specific problems such as wind loads on low-building flat roofs [27], wind loads on cars, lorries and trains travelling on bridges [28–30], dust spreading on cargo docks [31], or the oscillations of railway contact wires produced by galloping phenomena [32]. The results of these works indicate a positive effect of porous fences in terms of reduction of wind effects.

With regard to the general railway transport system, it should be said that cross-winds can strongly affect both railway infrastructure and rolling stock travelling along it. On the one hand, galloping phenomena have been reported to influence the safe operation of the railway system [33, 34]. On the other hand, the most damaging aerodynamic loads on trains are mainly determined by the cross-wind speed and the shape of both the vehicle and the surroundings [35]. The risk of train overturning increases if cross-wind speed reaches a threshold value. This threshold value is defined by the Characteristic Wind Curve (CWC) to provide a certain level of protection against train overturning [36]. In relation to the flow pattern around a train travelling under cross-wind, it should be pointed out that one of the most damaging aerodynamic effects in civil aerodynamics, the conical vortex [27], has been observed, both experimentally [37–39] and numerically [40], on the upper leeward corner of trains at certain yaw angles. As in the aforementioned cases regarding crops protection or noise and odour reduction, different types of parapets have been proposed to alleviate the effect of conical vortices, acting on their position with respect to the studied structure and, especially in the case of porous parapets, on their intensity as some small-scale turbulence generated at the parapets may interact with the vortices and reduce the generated suction on the structure surface [41]. Some efforts have been made to analyse the effectiveness of parapets and windbreaks to protect trains and other vehicles from cross-wind effects [42]. However, there seems to be a lack of qualitative and organised information regarding the shielding effects of wind protection devices placed around railway embankments. To the authors' knowledge, most of the studies focusing on train loads due to cross-winds at embankments have considered only the unprotected case [12, 35, 43]. Nevertheless, it is also fair to say that the protected case, with static and moving train models, has been studied in [44].

### 1.3. Aim of the Present Work

The aim of the present work is to analyse the influence of the windbreak geometry on the aerodynamic loads produced on trains and other rolling stocks on a railway embankment. The effect of straight windbreaks is compared to the effect of windbreaks equipped with different length eaves located at the tip. This effect of the parapet geometry has already been tested regarding building aerodynamics [45–47], with very good results in terms of wind-loads reduction when the parapets were equipped with eaves at their tip [41].

A 2-dimensional testing campaign was planned and carried out at the IDR/UPM laboratory, taking as the main comparison parameter the aerodynamic loads on a typical train section. Experimental results corresponding to the coach placed at both the windward and the leeward railway tracks are included in this work. Several models were built to reproduce a twin railway track with two different embankments, a set of solid windbreaks, and the coach model. The 2-dimensional experimental analysis should be considered a first approximation to the problem, as it is clear that the aerodynamic flow pattern around the leading car of a train is 3-dimensional once the train has reached a certain speed, especially if the aforementioned conical vortex is formed on the leading upper edge. However, it should also be mentioned that the fluid flow structure and the suction caused by this particular aerodynamic effect, that is, the conical vortex, have been successfully analysed with 2-dimensional models [48–50]. Furthermore, a similar tendency regarding the effects of parapets (in terms of wind-load reduction on roofs) when oblique and perpendicular-to-roof-edge wind flows are compared has been experimentally measured [51], indicating that the positive effect of the windbreak barrier is not only measured in the worst case (generally, in case of oblique wind direction), but also reflected in case of perpendicular-to-roof-edge wind directions.

In Section 2 of the present work the testing configuration and the facility (i.e., the wind tunnel) are described. The results are included and discussed in Section 3 and, finally, conclusions are summarized in Section 4.

## 2. Testing Configuration and Experimental Set-Up

The experimental set-up was planned and developed to analyse the aerodynamic loads on a coach surface in a 2-dimensional testing facility, when the train is placed at both the windward and the leeward railway tracks on an embankment model; see Figure 1. A 1/50 scale 2-dimensional model corresponding to an existing train manufactured by a Spanish enterprise has been reproduced. The coach model width and height are *c*_*c*_ = 59 mm and *h*_*c*_ = 82 mm, respectively. The distance from the top of the coach to the crest of the embankment is *h*_*d*_ = 102 mm. The distance from the edge of the embankment to the track middle point is *l*_*w*_ = 85 mm (windward track) and *l*_*l*_ = 195 mm (leeward track). The embankment slope vertical length is *h*_*S*_ = 80 mm. Two different horizontal lengths were considered for the embankment slope, *l*_*S*_ = 80 mm (1 : 1 slope) and *l*_*S*_ = 160 mm (1 : 2 slope). The twin railway track model length is *c* = 280 mm. The windbreak height, *h*, and the eave length, *a*, are indicated in the windward parapet sketched in Figure 1.

The coach was attached to the ballast with two rectangular prisms to simulate the distance between the track and the train model. Different static rolling angles of the coach were considered in order to determine its influence on the aerodynamic load coefficients induced by cross-wind. The definition of the rolling angle is represented in Figure 2. Three different values were considered, *β* = −6°, 0°, and 6°. The windbreak models tested consist of a solid vertical wall, 5 mm thick, placed on both edges of the embankment (see Figure 1) that can be equipped with different length eaves.

A first set of measurements were carried out with the train model located at the windward track, for the three rolling angles considered, and eight different straight (with no eave, that is, *a* = 0 mm) windbreaks heights, *h* = 0, 5, 10, 15, 25, 35, 45, and 55 mm in each case. After that, new measurements were taken for each of the three rolling angles considered, with *h* = 10, 15, 25, 35, 45, and 55 mm height windbreaks equipped with three different length eaves: *a* = 5, 10, and 15 mm. The aforementioned testing configurations were repeated with the train located at the leeward track. As previously mentioned, the wind tunnel tests have been carried out using two embankment slope ratios, 1 in 1 (1 : 1) and 1 in 2 (1 : 2). 312 different configurations were analysed. The complete testing configuration, equipped with an embankment slope 1 : 2, is shown in Figure 3. As it can be observed in the figure, the embankment slope consists of a triangular prism 80 mm high and wide enough to provide the considered slope.

The model configuration includes a *l*_*T*_ = 1600 mm spanned ground, slightly larger than the embankment width (*l*_*E*_ = *c* + 2*l*_*S*_), to ensure an appropriate simulation of the flow direction over the model; see Figures 1 and 3. The leading edge of this spanned ground is rounded in order to prevent boundary layer separation.

The model was equipped with 48 pressure taps along its middle section; see Figure 4 and Table 1. The pressure taps are made of 1 mm inner brass tubes connected to the pressure scanner through the pneumatic inputs. The pressure signal corresponding to each pressure tap is measured during 20 second, at 100 Hz sampling rate. The pressure coefficient, *c*_*p*_, is defined as

(1) $$\begin{array}{c} c_{p}\left(x,z\right)=\frac{p\left(x,z\right)-p_{s}}{q}, \end{array}$$

where *p*(*x*, *z*) is the averaged pressure measured at each pressure tap on the model surface (*x* and *z* stand for the pressure tap coordinates in a reference frame indicated in Figure 1; see also Table 1). The global aerodynamic coefficients are obtained by numerical integration of the pressure coefficients on the model surface, and they are expressed as

(2) $$\begin{array}{c} c_{d}=-\frac{1}{h_{c}}\oint c_{p}\left(x,z\right)\text{d}z,\\ c_{l}=-\frac{1}{h_{c}}\oint c_{p}\left(x,z\right)\text{d}x,\\ c_{m0}=-\frac{1}{h_{c}c_{c}}\left(-\oint z\cdot c_{p}\left(x,z\right)\text{d}z+\oint x\cdot c_{p}\left(x,z\right)\text{d}x\right),\\ c_{mv}=c_{m0}+c_{d}\cdot \frac{h_{c}}{2c_{c}}+c_{l}\frac{t}{2c_{c}}, \end{array}$$

where *c*_*d*_ is the side force coefficient, *c*_*l*_ is the lift coefficient, *c*_*m*0_ is the moment coefficient around the centre point of the model, *c*_*mv*_ is the moment coefficient around the leeward rail, *h*_*c*_ and *c*_*c*_ stand for the height and width of the coach, respectively, and *t* is the track width. Note that to simplify the numerical integration *c*_*m*0_ is calculated at the coach centre point, that is, the middle point of its symmetry line; see also Figure 1.

The IDR/UPM Institute A4C wind tunnel was used in this testing campaign; see Figure 5. This facility is an open-circuit wind tunnel with a closed test section that was used to perform a set of two-dimensional tests. The wind tunnel working section is 1.8 m high, 0.2 m wide, and 1.8 m long. A Scanivalve Corp. pressure scanner, model ZOC33, with 128 pressure inputs, has been used to measure the pressure on the model surface. An Airflow pitot tube is used to determine the dynamic pressure, *q*, as *q* = *p*_0_ − *p*_*S*_ = *ρU*_*∞*_^2^/2, where *p*_0_ is the stagnation pressure, *p*_*s*_ is the static pressure of the upstream flow, and *ρ* stands for the air density and *U*_*∞*_ is the free flow velocity. Measurements were done at *U*_*∞*_ = 22 m/s wind speed, with 5.5% turbulence intensity. The tests are carried out placing the model at the centre of the testing chamber, with a 1 mm gap being left between the model and the chamber walls. As is well known, the size of the working section establishes a maximum admissible size of the model in order to ensure proper boundary conditions [52–54]. In order to minimize the blockage effects as much as possible, the scale 1/50 was chosen.

The studied configurations were tested in low turbulence conditions. The rolling moment of trains due to wind loads has already been analysed in such condition [13, 40, 55], and although experiments under low turbulence condition produce some differences compared to the results from tests carried out with wind boundary layer simulation, it should also be mentioned that the general flow pattern is not altered, the rolling moment being very similar. For instance, Cheli et al. [55] show the rolling moment coefficient on a van vehicle as a function of the wind yaw angle, measured in low turbulence conditions and with wind boundary layer simulation (see Figure 6). It can be appreciated in that figure that, leaving aside some slight differences, the results are essentially similar.

## 3. Results and Discussion

As stated in Section 2, 312 different configurations were measured. In Figures 7, 8, 9, and 10 the pressure coefficient plotted for all rolling angles and both embankment slopes are shown as a function of the nondimensional distance over the train surface, *s*/*s*_max⁡_, defined in Figure 4 (obviously, *s*/*s*_max⁡_ = 0.5 at the top of the train, *s*/*s*_max⁡_ < 0.5 being the windward surface and *s*/*s*_max⁡_ > 0.5 the leeward surface). Only cases corresponding to eave lengths *a* = 0 mm and *a* = 10 mm have been included in Figures 7–10, as small variations regarding eave length at the tip of the windbreaks seem to have negligible effects on the force coefficients. In Table 2 these force coefficients, *c*_*l*0_, *c*_*d*0_, and *c*_*mv*0_, corresponding to all configurations tested without parapets, are included. As mentioned, these coefficients were calculated based on the pressure distributions measured on the train surface (expressions (2)).

As expected, side force and rolling moment decrease when the train is located on the leeward track for both slopes tested. The reduction is around Δ*c*_*d*0_ = −55% and Δ*c*_*mv*0_ = −44% with respect to the train on the windward track, for rolling angles *β* = 0° and *β* = 6°. In the case of a negative rolling angle, *β* = −6°, the reduction with regard to the side force is similar to the aforementioned one, Δ*c*_*d*0_ = −53% (slope 2 : 1) and Δ*c*_*d*0_ = −58% (slope 1 : 1); however, there is a significant variation on the figures regarding the reduction of the rolling moment, Δ*c*_*mv*0_ = −26% (slope 2 : 1) and Δ*c*_*mv*0_ = −16% (slope 1 : 1). The explanation for this effect can be found if the lift coefficients are analysed. Despite lift coefficients corresponding to rolling angles *β* = 0° and *β* = 6° being quite similar (although the train located at the leeward track is exposed to higher lift forces), a big change is observed comparing the lift coefficients at *β* = 0° and *β* = −6°. The variation is quite large, with even a change of the lift force direction, in the case of the train located at the windward track for both tested embankment slopes. These changes are due to the variation of the pressure coefficient distribution on the train surface. A great suction at the lower part of the windward surface, with a peak close to *s*/*s*_max⁡_ = 0.05, is produced by the wind for *β* = −6° when the train is located at the windward track for both tested slopes (see Figures 7 and 9). This suction is created by the acceleration of the flow under the train due to the negative rolling angle. The negative rolling angle configuration produces a lower stagnation point at the train windward surface, increasing the Venturi effect under the train, and therefore the lift is reduced when compared to the *β* = 0° configuration.

In order to study the effect of the tested windbreaks, the nondimensional lift (*c*_*l*_/*c*_*l*0_), side force (*c*_*d*_/*c*_*d*0_), and rolling moment (*c*_*mv*_/*c*_*mv*0_) coefficients calculated from the measured pressure distributions are shown in Figure 11 (slope 1 : 2; windward track), Figure 12 (slope 1 : 2; leeward track), Figure 13 (slope 1 : 1; windward track), and Figure 14 (slope 1 : 1; leeward track), as a function of the dimensionless height of the windbreak, *h*/*h*_*d*_ (the height of the train over the ground, *h*_*d*_, was chosen as a logical reference; see Figure 1).

The results included in the mentioned figures were made dimensionless with the values of lift, side force, and rolling moment coefficients (*c*_*l*0_, *c*_*d*0_, and *c*_*mv*0_) resulting from the case measured with no windbreak installed and *β* = 0° rolling angle. Obviously, due to the train cross-section and the configurations analysed, there seems to be a greater correlation between the rolling moment coefficient and the side force coefficient than between the rolling moment and the lift. It can be observed in the figures that the eaves at the tip of the windbreak do have a considerable effect on the pressure distribution and consequently on the force coefficients, although, as said, the effect of the eave length does not seem to be significant (force coefficients from the same windbreak heights and different eave length are very similar). Also, the results from the same windbreak and track configurations, but with changing the embankment slope, indicate a reduced effect of this parameter.

Focusing on the case of the train located on the windward track, an increase of the lift coefficient, *c*_*l*_/*c*_*l*0_, is shown in most of the cases for low values of *h*/*h*_*d*_. Then, as the height of the windbreak increases, the lift coefficient ratio decreases to negligible values for the higher windbreaks tested (see Figures 11 and 13). The variations in the lift coefficient are a direct consequence of changes in the intensity of the suction peak located on the coach roof surface. Initially, as the parapet height increases, the intensity of the suction peak increases as the velocity of the flow is rising close to the round upper corner of the train, and the stagnation point is closer to this corner. However, for *h*/*h*_*d*_ = 0.34 and higher heights, the pressure distribution is more uniform, the suction peak being reduced. This reduction on the wind suction is probably caused by the shear layer created at the upper extreme of the windbreak, which introduces small-scale turbulence on the flow close to the mentioned round upper corner (increasing the wind-flow turbulence over low-rise building roofs sheltered by solid parapets has turned into a similar reduction on the mean suctions measured on the aforementioned roofs [27]).

Side force coefficient, *c*_*d*_/*c*_*d*0_, shows a more uniform trend in all the cases, with the exception of windbreaks without eave and positive rolling angles of the train. As already mentioned, the results from Figures 7–10 indicate that pressure distribution becomes more uniform with the windbreak height. Consequently, side force coefficient ratio decreases as the windbreak height increases. In fact, if the windbreak height is large enough the side force coefficient becomes negative; that is, the aerodynamic force on the coach is acting against the main direction of the incident flow. This effect is in accordance with former studies on the wind loads on the leeward windbreak installed on similar emplacements (cliffs and embankments) provided with wind protection devices [56]. Similar effects have been reported in the side force of buildings placed inside the wake of buildings with similar geometric characteristics [57, 58]. More specifically related to the wind-train interaction, it should be mentioned that this effect has already been reported for both static and moving model tests [44], the recirculating flow pattern in the separation bubble behind the fence being suggested as presumably the main cause of this behaviour.

Regarding the rolling moment coefficient, *c*_*mv*_/*c*_*mv*0_, the trend is quite similar to the one shown by the side force coefficient ratio, with a change of the direction for the higher windbreaks. Furthermore, it should be pointed out that significant values of this reversed rolling moment were measured for the higher windbreaks tested. This effect indicates the important role of the aerodynamic side force in the lateral equilibrium of the vehicle.

The trends shown by the aerodynamic force coefficients corresponding to the train located on the leeward track are more uniform, in contrast to the mentioned ones regarding the train at the windward track; see Figures 12 and 14. In the configurations corresponding to the train at this position, all the lift coefficients, *c*_*l*_/*c*_*l*0_, smoothly decrease as the windbreak height increases. As can be observed in Figures 7–10, an appreciable suction peak appears on the train roof surface when no windbreaks are installed. As the windbreak height increases the area enclosed by the suction peak decreases and, as a result, the lift coefficient decreases, being negligible for the higher windbreaks tested. The behaviour of the side force coefficient, *c*_*d*_/*c*_*d*0_, as a function of the windbreak height has a similar pattern to the ones measured in the windward configurations. When the windbreak reaches a certain height the side force on the train opposes the upstream flow direction. Besides, as in the studied windward configurations, the rolling moment coefficient, *c*_*mv*_/*c*_*mv*0_, shows similar trends to the ones from the side force coefficient, *c*_*d*_/*c*_*d*0_.

In order to extract more practical information from the results, the values of the percentage reduction obtained using the wind eaves in relation to the aerodynamic force/rolling moment coefficient corresponding to the case of windbreak 6 without any eave (*a* = 0),

(3) $$\begin{array}{c} \Delta \frac{c_{l}}{c_{l0}}=\frac{{\left.c_{l}/c_{l0}\right|}_{a=0}-{\left.c_{l}/c_{l0}\right|}_{a}}{{\left.c_{l}/c_{l0}\right|}_{a=0}},\\ \Delta \frac{c_{d}}{c_{d0}}=\frac{{\left.c_{d}/c_{d0}\right|}_{a=0}-{\left.c_{d}/c_{d0}\right|}_{a}}{{\left.c_{d}/c_{d0}\right|}_{a=0}},\\ \Delta \frac{c_{mv}}{c_{mv0}}=\frac{{\left.c_{mv}/c_{mv0}\right|}_{a=0}-{\left.c_{mv}/c_{mv0}\right|}_{a}}{{\left.c_{mv}/c_{mv0}\right|}_{a=0}}, \end{array}$$

are shown in Table 3. Obviously, the data from the train located at windward track is reflected in the table, as the effects of the eaves on the aerodynamic loads are much lower when the train is located at leeward track. The summarized results included in Table 3 show a quite remarkable reduction of the aerodynamic loads when an eave is added to the parapet. This is not really surprising, as other studies have shown an increase of the wind-load reduction reached with parapets equipped with an extra shape characteristic which make then non-just-vertical-solid parapets. As an example, with these non-vertical-solid parapets (porous parapets, cantilever parapets, etc.) the wind loads on building roofs have been reduced by up to 50%–70% [27, 41, 46], these figures being similar to the maximum ones resulting from the present work (see Table 3). Finally, it should be pointed out that the proposed eaves represent a new configuration that could be considered an easy and cheap way to increase the effectiveness of the solid parapets in terms of aerodynamic load reduction.

## 4. Conclusions

In the present study the windbreak sheltering effect on the cross wind-flow around a train (rolling-stock) is experimentally analysed, taking the pressure distribution and the aerodynamic force coefficients (lift, side force, and rolling moment) as the main comparison parameters. Two different embankments, 1 : 2 and 1 : 1 slopes, are studied, together with three rolling angle positions, *β* = −6°, 0°, and 6°. The major conclusions resulting from this work are as follows.

- Windbreaks, even those with small heights, provide sheltering effects to the vehicle. For the most exposed-to-the-wind configuration (windward track and 1 : 2 embankment, see Table 2), the smaller-height windbreaks (*h*/*h*_*d*_ = 0.049) produced a reduction of 34% (*β* = −6°), 52% (*β* = 0°), and 6% (*β* = 6°), with regard to the measured rolling moment coefficients.
- If the windbreak is high enough (*h*/*h*_*d*_ ~ 0.2-0.3), side force and rolling moment coefficients become reversed.
- As expected, results indicate that the side force is the main influence on the overturning moment.
- The shielding effect of the windbreaks is improved when an eave is installed at their tips. However, the influence of the eave length seems to be negligible to some extent, at least amongst the tested eave lengths.

## Figures and Tables

**Figure 1:** Sketch of the tested configuration: embankment and the twin railway track model equipped with windbreaks. Coefficients *c*_*l*_, *c*_*d*_, and *c*_*mv*_ (lift, side force, and rolling moment) are also indicated.

**Figure 2:** Coach rolling angle, *β*. Negative values of the rolling angle correspond to a counterclockwise rotation around *y*-axis (a), whereas positive values correspond to a clockwise rotation around *y*-axis (b).

**Figure 3:** Sketch of the embankment model and the twin railway track equipped with windbreaks. The train coach model is located on the windward rail track. The embankment slope vertical length is *h*_*S*_ = 80 mm. The length of the embankment is *l*_*E*_ = *c* + 2*l*_*S*_. The width and length of the complete mock-up are *w* = 200 mm and *l*_*T*_ = 1600 mm, respectively.

**Figure 4:** Coach/train model used for the two-dimensional tests during the pressure measurement campaign (a). The nondimensional distance over the train surface at the middle cross-section, *s*/*s*_max⁡_, is indicated (b).

**Figure 5:** A4C wind tunnel. Isometric view (a) and top view (b): 1—nozzle with two-dimensional contraction, 2—test section, 3—diffuser, 4—centrifugal fans, 5—open flow return, 6—test section access door, 7—instrumentation and technical equipment, and 8—power control system.

**Figure 6:** Low turbulence versus mean turbulence effect on the rolling moment coefficient, *c*_*mx*_, on a lorry reported by Cheli et al. [55]. Rolling moment coefficient measured as a function of the yawing angle, *α* (a); and pressure coefficients measured on the surface of the lorry (van and truck) at *α* = 90° (b). Low and mean turbulence wind profiles are also indicated in the sketch on the right side.

**Figure 7:** Pressure coefficient, *c*_*p*_, distributions with the coach placed on the windward railway track on an embankment with a slope 1 : 2, as a function of the nondimensional distance over the train surface at the middle cross-section, *s*/*s*_max⁡_ (see Figure 4(b)).

**Figure 8:** Pressure coefficient, *c*_*p*_, distributions with the coach placed on the leeward railway track on an embankment with a slope 1 : 2, as a function of the nondimensional distance over the train surface at the middle cross-section, *s*/*s*_max⁡_ (see Figure 4(b)).

**Figure 9:** Pressure coefficient, *c*_*p*_, distributions with the coach placed on the windward railway track on an embankment with a slope 1 : 1, as a function of the nondimensional distance over the train surface at the middle cross-section, *s*/*s*_max⁡_ (see Figure 4(b)).

**Figure 10:** Pressure coefficient, *c*_*p*_, distributions with the coach placed on the leeward railway track on an embankment with a slope 1 : 1, as a function of the nondimensional distance over the train surface at the middle cross-section, *s*/*s*_max⁡_ (see Figure 4(b)).

**Figure 11:** Lift, *c*_*l*_/*c*_*l*0_, side force, *c*_*d*_/*c*_*d*0_, and rolling moment, *c*_*mv*_/*c*_*mv*0_, coefficient ratios as a function of the windbreak height, when the train coach is placed on the windward rail on the embankment with slope 1 : 2. Four eave lengths are considered, *a* = 0 mm (circles), *a* = 5 mm (rhombi), *a* = 10 mm (squares), and *a* = 15 mm (triangles). Each column represents a different coach rolling angle, *β* = −6° (left), *β* = 0° (centre), and *β* = 6° (right).

**Figure 12:** Lift, *c*_*l*_/*c*_*l*0_, side force, *c*_*d*_/*c*_*d*0_, and rolling moment, *c*_*mv*_/*c*_*mv*0_, coefficient ratios as a function of the windbreak height, when the train coach is placed on the leeward rail on the embankment with slope 1 : 2. Four eave lengths are considered, *a* = 0 mm (circles), *a* = 5 mm (rhombi), *a* = 10 mm (squares), and *a* = 15 mm (triangles). Each column represents a different coach rolling angle, *β* = −6° (left), *β* = 0° (centre), and *β* = 6° (right).

**Figure 13:** Lift, *c*_*l*_/*c*_*l*0_, side force, *c*_*d*_/*c*_*d*0_, and rolling moment, *c*_*mv*_/*c*_*mv*0_, coefficient ratios as a function of the windbreak height, when the train coach is placed on the windward rail on the embankment with slope 1 : 1. Four eave lengths are considered, *a* = 0 mm (circles), *a* = 5 mm (rhombi), *a* = 10 mm (squares), and *a* = 15 mm (triangles). Each column represents a different coach rolling angle, *β* = −6° (left), *β* = 0° (centre), and *β* = 6° (right).

**Figure 14:** Lift, *c*_*l*_/*c*_*l*0_, side force, *c*_*d*_/*c*_*d*0_, and rolling moment, *c*_*mv*_/*c*_*mv*0_, coefficient ratios as a function of the windbreak height, when the train coach is placed on the leeward rail on the embankment with slope 1 : 1. Four eave lengths are considered, *a* = 0 mm (circles), *a* = 5 mm (rhombi), *a* = 10 mm (squares), and *a* = 15 mm (triangles). Each column represents a different coach rolling angle, *β* = −6° (left), *β* = 0° (centre), and *β* = 6° (right).

**Table 1:** Nondimensional coordinates regarding each pressure tap installed on the model surface. The reference axes are shown in Figures 1 and 4.

Pressure tap	*x*/*h*	*y*/*h*	*s*/*s*_max⁡_
1	0.00	0.50	0.50
2	−0.06	0.50	0.48
3	−0.12	0.49	0.46
4	−0.18	0.47	0.44
5	−0.23	0.45	0.42
6	−0.28	0.40	0.40
7	−0.31	0.35	0.37
8	−0.33	0.28	0.35
9	−0.35	0.22	0.33
10	−0.35	0.16	0.31
11	−0.35	0.10	0.29
12	−0.36	0.04	0.27
13	−0.36	−0.02	0.25
14	−0.36	−0.08	0.23
15	−0.36	−0.14	0.21
16	−0.36	−0.21	0.19
17	−0.35	−0.27	0.16
18	−0.34	−0.33	0.14
19	−0.31	−0.39	0.12
20	−0.29	−0.45	0.10
21	−0.24	−0.48	0.08
22	−0.19	−0.49	0.06
23	−0.13	−0.49	0.04
24	−0.06	−0.50	0.02
25	0.00	−0.50	0.00
26	0.06	−0.50	0.98
27	0.13	−0.49	0.96
28	0.19	−0.49	0.94
29	0.24	−0.48	0.92
30	0.29	−0.45	0.90
31	0.31	−0.39	0.88
32	0.34	−0.33	0.86
33	0.35	−0.27	0.84
34	0.36	−0.21	0.81
35	0.36	−0.14	0.79
36	0.36	−0.08	0.77
37	0.36	−0.02	0.75
38	0.36	0.04	0.73
39	0.35	0.10	0.71
40	0.35	0.16	0.69
41	0.35	0.22	0.67
42	0.33	0.28	0.65
43	0.31	0.35	0.63
44	0.28	0.40	0.60
45	0.23	0.45	0.58
46	0.18	0.47	0.56
47	0.12	0.49	0.54
48	0.06	0.50	0.52

**Table 2:** Force coefficients, *c*_*l*0_, *c*_*d*0_, and *c*_*mv*0_, corresponding to the configurations tested without parapets (*h* = 0). The reference axes are shown in Figure 1.

Train at windward track				Train at leeward track			
*β* [°]	*c*_*l*0_	*c*_*d*0_	*c*_*mv*0_	*β* [°]	*c*_*l*0_	*c*_*d*0_	*c*_*mv*0_
Embankment slope 1 : 2							
−6	−0.27	1.26	0.47	−6	0.58	0.53	0.35
0	0.31	1.24	0.65	0	0.91	0.54	0.38
6	0.29	1.27	0.65	6	1.03	0.59	0.35

Train at windward track				Train at leeward track			
*β* [°]	*c*_*l*0_	*c*_*d*0_	*c*_*mv*0_	*β* [°]	*c*_*l*0_	*c*_*d*0_	*c*_*mv*0_

Embankment slope 1 : 1							
−6	−0.17	1.18	0.45	−6	0.57	0.56	0.38
0	0.29	1.21	0.63	0	0.82	0.48	0.35
6	0.24	1.25	0.63	6	0.99	0.57	0.35

**Table 3:** Highest percentage reduction on the aerodynamic loads on the train at windward track with eave-parapets, in relation to the aerodynamic loads measured with no-eave-parapets (*a* = 0). The height of the parapet where the highest reduction is obtained is also included in each case.

*β* [°]	*a* [mm]	Δ*c*_*l*_/*c*_*l*0_	*h*/*h*_*d*_	Δ*c*_*d*_/*c*_*d*0_	*h*/*h*_*d*_	Δ*c*_*mv*_/*c*_*mv*0_	*h*/*h*_*d*_

Embankment slope 1 : 2 (train at windward track)							
−6	5	6.9%	0.15	36.9%	0.15	12.9%	0.10
	10	13.1%	0.15	39.4%	0.15	15.4%	0.10
	15	17.1%	0.15	39.0%	0.15	16.3%	0.10

0	5	10.8%	0.15	17.8%	0.10	4.0%	0.10
	10	16.0%	0.15	21.3%	0.54	5.2%	0.34
	15	2.3%	0.10	20.9%	0.54	9.5%	0.10

6	5	21.8%	0.25	1.4%	0.54	36.1%	0.10
	10	21.5%	0.25	55.6%	0.10	20.6%	0.34
	15	30.0%	0.25	63.3%	0.10	24.8%	0.34

*β* [°]	*a* [mm]	Δ*c*_*l*_/*c*_*l*0_	*h*/*h*_*d*_	Δ*c*_*d*_/*c*_*d*0_	*h*/*h*_*d*_	Δ*c*_*mv*_/*c*_*mv*0_	*h*/*h*_*d*_

Embankment slope 1 : 1 (train at windward track)							
−6	5	8.7%	0.15	3.0%	0.54	3.4%	0.54
	10	12.3%	0.15	37.7%	0.15	12.1%	0.15
	15	6.3%	0.10	33.7%	0.15	11.2%	0.15

0	5	11.8%	0.10	9.5%	0.54	10.4%	0.54
	10	18.3%	0.10	4.2%	0.25	16.3%	0.54
	15	21.7%	0.10	12.5%	0.54	13.0%	0.54

6	5	27.0%	0.25	67.9%	0.10	55.6%	0.15
	10	36.5%	0.25	75.7%	0.15	60.8%	0.15
	15	39.7%	0.25	65.9%	0.25	58.0%	0.15
